The article "Application of Ultrasound-Guided Upper Trunk Brachial Plexus Block in Observation of Lower Shoulder Surgery" was retracted in 2023. Reasons: signs of a paper mill; suspected computer-generated content; unreliable results or conclusions; lack of ethics approval or compliance.

# Application of Ultrasound-Guided Upper Trunk Brachial Plexus Block in Observation of Lower Shoulder Surgery

**DOI:** 10.1155/2022/9168566

**Published:** 2022-06-27

**Authors:** Dehua Yu, Jingjing Jiang, Zongming Jiang, Zhonghua Chen, Qifu Zhou

**Affiliations:** Department of Anesthesiology, Shaoxing People's Hospital Shaoxing Hospital, Zhejiang University School of Medicine, Shaoxing, Zhejiang 312000, China

## Abstract

This study aims to ensure the wide application of ultrasound-guided superior brachial plexus block in shoulder surgery, solve the application problem of ultrasound-guided superior brachial plexus block in shoulder surgery, make up for severe postoperative pain after shoulder arthroscopy, and improve the patient's recovery ability. In this paper, 90 patients with shoulder arthroscopy were divided into 3 groups: A, B, and C. In recent years, with the rapid development of medicine, ultrasound-guided brachial plexus upper trunk block has been widely used in shoulder surgery. Shoulder arthroscopy is more and more used in the diagnosis and treatment of shoulder diseases because of its advantages of minimally invasive, safe, and rapid recovery. Compared with the traditional operation, it is found that the shoulder arthroscopic operation reduces the incision trauma through the microscope, but the shoulder operation involves more muscles and ligaments, so the perioperative pain of shoulder arthroscopic operation is still serious.

## 1. Introduction

Due to the narrow operation area of shoulder arthroscopy, in order to clarify the operation field, it is necessary to apply pressurized articular cavity flushing and controlled hypotension technology in order to control the bleeding in the operation field. Coupled with the influence of body position, perioperative pain management, intraoperative hemodynamic management, and rapid rehabilitation of postoperative patients all put forward new requirements for anesthesiologists [1]. In shoulder surgery patients, the use of ultrasound-guided intercostal space combined with upper thoracic obstruction and general anesthesia can not only provide preoperative analgesia, but also reduce the dose of general anesthesia drugs, shorten the recovery time of patients, facilitate the implementation of controlled hypotension, and make the hemodynamics of patients more stable during operation. On this basis, ultrasound-guided upper trunk block of brachial plexus reduced the impact on elbow flexion and wrist flexion and improved the satisfaction of patients.

The shoulder joint is reinforced by the following ligaments: The coracobrachialis ligament strengthens the upper part of the joint capsule and has the functions of limiting the lateral rotation of the humerus and preventing the upward dislocation of the humeral head. The glenohumeral ligament is on the front wall of the joint capsule, which can strengthen the front wall of the joint capsule. The transverse ligament of the humerus is the inherent ligament of the humerus, which plays the role of fixing the tendon of the long head of the biceps brachii in the tubercular sulcus [2, 3], as shown in Figure 1.

Arthroscopic shoulder surgery is less invasive and safer than traditional open shoulder surgery. Shoulder arthroscopy requires lateral positioning, irrigation of the joint cavity, and control of hypotension; it may affect the patient's breathing. Therefore, general anesthesia is the main method for shoulder arthroscopy. With the deepening of the research on the mechanism of pain, the application of nerve block in shoulder arthroscopic surgery is gradually increasing. The postoperative blood flow, anesthesia dose, and postoperative recovery quality were compared between simple general anesthesia and ultrasound-guided general anesthesia for superficial trunk and neck obstruction in shoulder arthroscopy. In order to provide reference for improving the anesthesia quality of shoulder arthroscopic surgery, this paper compared the application of general anesthesia combined with upper trunk brachial plexus and superficial cervical plexus nerve block in shoulder arthroscopic surgery from the aspects of intraoperative circulation, anesthetic drug dosage, and postoperative recovery quality [4].

## 2. Literature Review

According to Sahara, R., like others, general anesthesia is the most commonly used anesthesia in laparoscopic shoulder surgery [5]. In order to obtain a clear visual field under the microscope, continuous pressure flushing in the articular cavity and intraoperative controlled hypotension are needed in shoulder arthroscopy. Intraoperative intra-articular pressure irrigation can easily cause tracheal mucosal edema and neck tissue edema, compress the trachea, and lead to upper respiratory tract obstruction and even asphyxia. Chen, G. believed that when general anesthesia was adopted for endotracheal intubation, it was convenient for respiratory management and ensured the oxygen supply and ventilation during operation [6]. Yakovenko, S. believed that general anesthesia can eliminate the blood pressure fluctuation caused by patients' emotional tension and is also conducive to the implementation of controlled hypotension [7]. At the same time, the dosage is accurate, with the advantages of high safety and convenient operation. However, the recovery time after general anesthesia is relatively long, resulting in high anesthesia risk and high incidence of complications after anesthesia. Qiang, L. believed that regional block anesthesia was simple and safe with few complications [8]. Lee, K. said that the anesthesia method does not affect the patient's state of consciousness, has little impact on other physiological functions, and still has analgesic effect after operation, which is helpful for the patient to start functional exercise early [9].The current regional nerve block methods used for shoulder arthroscopic surgery are intermuscular sulcus, bronchial block, upper trunk block, superior cervical nerve block, and axillary nerve block. According to Meder, A., brachial plexus block is a commonly used anesthetic in endoscopic shoulder surgery. It relaxes muscles during surgery, provides analgesia, and provides good postoperative analgesia [10]. At the same time, the dosage of surgical anesthetics and postoperative analgesics can be reduced, and the side effects of nausea and vomiting can be reduced. It has been reported that brachial plexus block can shorten the stay time and hospital stay of patients undergoing shoulder arthroscopic surgery in the anesthesia recovery room. The traditional block method is located by anatomical body surface markers, sense of vision method, and nerve stimulator. The operation time of block is long, and the number of punctures is more. The application of ultrasound-guided technology in nerve block greatly shortens the operation time, reduces the number of punctures, and enhances the blocking effect.

N., N. believed that ISBB and SCBB have been used for anesthesia in shoulder surgery [11]. Some viewpoints believe that compared with ISBB, SCBB can also achieve good results in postoperative analgesia and postoperative recovery after shoulder arthroscopic surgery, and its blocking site is far away from the phrenic nerve, which can reduce the incidence of hemi-phrenic nerve paralysis. However, SCBB is generally considered ineffective in blocking the suprascapular nerve. The suprascapular nerve arises from the C5 and C6 nerve roots of the superior tracheal trunk and sometimes from C4. It regulates the movement of the shoulder joint capsule, the acromioclavicular joint, the subacromial tubercle capsule, the posterior coracoclavicular tendon, and the upper and lower spinal muscles. Incomplete occlusion of the suprascapular nerve results in pain relief. Research by Chen, S. et al. proves just that. Therefore, SCBB is not widely used in shoulder surgery [12]. Chen, S. and others proposed that SSNB combined with ANB is a safe and effective anesthesia method for shoulder arthroscopic surgery from the aspects of safety, intraoperative and postoperative analgesic effect, and patient satisfaction [13]. The injection position of this method is also far away from the respiratory related nerves (phrenic nerve and recurrent laryngeal nerve) in anatomy. Therefore, it is considered that it has less impact on respiratory function and can improve the insufficient analgesia of SSNB. However, this method is relatively difficult to operate and has high requirements for operators.

## 3. Method

### 3.1. Experiment

90 patients with ASA grade I ∼ II before anesthesia were selected for shoulder arthroscopic surgery. Rotator cuff injury was diagnosed before operation [14]. The cases were randomly divided into three groups, 30 cases in each group: group A was the general anesthesia control group; group B was the obstruction of the brachial plexus groove between the conventional muscles of ultrasound combined with general anesthesia; group C was a general anesthesia group with modified upper trunk brachial plexus and superficial cervical plexus nerve block under ultrasound guidance. Both groups were treated with 0.35% ropivacaine solution to relieve local nerve block. The changes of MAP and HR indexes before operation (T0), 5 minutes after operation (T1), 30 minutes after operation (T2), and 30 minutes after laryngeal mask removal (T3) were observed and recorded. The BIS value of the three groups remained between 45 and 60 during operation. We observed and recorded the BIS value and operation duration of patients 5 minutes (T1) and 30 minutes (T2) after the operation, the time of laryngeal mask removal after the operation (the time from sevoflurane withdrawal to laryngeal mask removal), and the dosage of opioid analgesics (sufentanil) and sevoflurane during the operation. The VAS scores of patients entering PACU, 6 h and 12 h after operation, and the muscle strength grades of elbow flexion and wrist flexion were observed and recorded. We observed and recorded the dosage of analgesic drugs and the occurrence of adverse reactions such as nausea, vomiting, vertigo, and respiratory depression 6 hours after operation [15].

Since the beginning of the twenty-first century, ultrasound technology has been more and more widely used in anesthesia. Before anesthesia, ultrasound imaging can quickly evaluate the patient's gastric volume, judge whether the patient's fasting time meets the specified standard, and avoid reflux and aspiration during operation. In spinal anesthesia and nerve block anesthesia, the application of ultrasonic visualization operation not only improves the success rate of anesthesia puncture, but also reduces the incidence of anesthesia complications. Different from the traditional anatomical localization method, ultrasound-guided nerve block has better effect, faster onset, and longer analgesic time and significantly reduces the incidence of related complications. Therefore, ultrasonic visualization technology has obvious advantages in nerve block anesthesia [16].

There were 90 patients, male and female. Inclusion criteria were as follows: (1) preoperative diagnosis of rotator cuff tear; (2) shoulder arthroscopic rotator cuff repair performed at a selected time; (3) age: 45 ∼ 75 years; (4) unilateral operation; (5) ASA class I ∼ II; (6) no history of cardiopulmonary and mental illness; (7) normal blood coagulation and liver and kidney function.

Ninety patients who were going to undergo laparoscopic shoulder surgery were randomly divided into three groups, 30 cases in each group:

1. Patients in group A received general anesthesia.
2. Patients in group B were treated with traditional intramuscular brachial plexus groove block under general anesthesia under ultrasound supervision. After entering the room, the patient was observed for 10 minutes, and 10 mL of 0.3% ropivacaine was injected around the muscle cyanosis. After the effect of the nerve block was determined, general anesthesia was administered.
3. Patients in group C received combined general anesthesia with modified upper trunk brachial plexus and superficial cervical plexus nerve block under ultrasound, and the superficial block of the upper trunk and cervical spine was modified. 7 ml and 5 ml of 0.35% ropivacaine were injected around the superior bronchial nerve and superficial cervical lymph nodes, respectively, with 10-minute observation. After the effect of the nerve block was determined, general anesthesia was administered.

After the patient entered the operating room, the upper limb intravenous access was opened, and sodium lactate Ringer's solution was injected to maintain body fluid balance. ECG, noninvasive cuff blood pressure, and pulse oximetry (SpO2) were regularly monitored, and oxygen was inhaled through a mask. After intravenous midazolam sedation, the contralateral radial artery was punctured and catheterized to monitor blood pressure. The blood pressure and heart rate measured after resting and 5 minutes were the blood pressure and heart rate at T0, and then nerve block was performed [17].

Sono-Turbo portable color ultrasound was used for nerve block. After the patient lies on a pillow, they turn their head to the healthy side for about 60 minutes. A 12 MHz ultrasound transducer is placed on the patient's neck to locate the internal carotid artery and vein. After taking cross-sectional images of the internal carotid artery and vein, the ultrasound probe is moved until it reaches the sternocleidomastoid muscle, and the tubular node is located and identified beneath it. Under ultrasound, the brachial plexus is imaged between the muscles in the front and middle of the neck. The brachial plexus image consists of three circular or oval hypoechoic areas; they are the upper body of the trachea, the middle body of the intervertebral disc, and the lower body of the major limbs. Then, the ultrasonic probe is slid to the lateral edge of the midpoint of the sternocleidomastoid muscle to find the prevertebral fascia. The prevertebral fascia under ultrasound is located on the surface of the intermuscular sulcus, and the superficial cervical plexus is close to the lower part of the prevertebral fascia. When the upper trunk of brachial plexus, the transverse section of sternocleidomastoid muscle, and the image of prevertebral fascia are on the same display screen, the ultrasonic probe is fixed [18].

After the nerve block effect is determined, sufentanil 0.3–0.4 mg/kg, propofol 2 mg/kg, and cisatracurium 0.2 mg/kg are given intravenously for general anesthesia. After using the tube mask, the anesthesia device is connected and IPPV is performed. The tidal volume is 6–8 ml/kg, the respiratory rate is 12 times/min, and the breath-to-breath ratio is 1 : 2. The respiratory parameters are adjusted, and the end expiratory carbon dioxide is maintained between 35 and 40 mmHg. Sevoflurane was inhaled continuously during the operation to maintain anesthesia. According to the intraoperative blood pressure and the depth of anesthesia, sufentanil 0.1 ug/kg and CIS atracurium 0.1 mg/kg were given intravenously. The BIS value of anesthesia depth was maintained between 45 and 60.

Intraoperative rehydration was 250 ml normal saline and 500 ml sodium lactate Ringer's solution. After the operation, MAP was maintained at 60 ∼ 80 mmHg. When MAP >80 mmHg, anesthetic drugs shall be added according to the intraoperative conditions; when MAP <60 mmHg, ephedrine shall be given appropriately to raise blood pressure. Inhalation of sevoflurane was stopped when the arthroscopy was completed and the wound was sutured [19]. Laryngeal mask removal criteria are as follows: the patient being awake; no obvious edema in head, neck, or upper limbs; spontaneous breathing tidal volume > 5 ml/kg, swallowing reflex recovery, and spontaneous lifting time > 5 s. Patients with HR < 50 times/min were given atropine symptomatic treatmentas needed.

There were no significant differences in age, gender, BMI, operation time, and BIS value between the three groups (*P* > 0.05).  Table 1 shows the comparison of the general conditionsand BIS valuesof the patients in each group.

1. At T0, there was no significant difference between the groups; compared with group A, the morphology of patients in other groups at T1, T2, and T3 was significantly reduced (*P*<0.05). The mean arterial pressure (figure) comparison of patients in each group is shown in Table 2 and Figure 2.
2. At T0, there was no significant difference between the groups; compared with group A, the HRs of patients in other groups at T1, T2, and T3 groups were significantly lower (*P*<0.05). The heart rate (HR) comparison of patients in each group is shown in Table 3 and Figure 3.

## 4. Results and Analysis

In surgery, the concept of minimally invasive surgery has become more and more advanced. With the continuous maturity of endoscopic operation, shoulder arthroscopic surgery (ASS) has been widely used in shoulder joint examination and rotator cuff injury treatment [20]. Arthroscopic shoulder surgery has the advantages of less trauma, less infection, and rapid rehabilitation. At present, it has gradually replaced open shoulder surgery.

When patients undergo shoulder arthroscopic surgery, they often use lateral position, and intra-articular pressure flushing is required during the operation, which may cause tissue edema and airway obstruction. Moreover, due to the special position of the shoulder joint, it is impossible to apply a tourniquet. Controlled hypotension is required during the operation to reduce the amount of bleeding and flushing fluid. Therefore, general anesthesia (GA) is preferred during the operation. Although general anesthesia alone has the advantages of definite effect and easy management of respiratory tract during operation, it cannot reduce the stress response of patients during operation. In addition, the dosage of anesthetic during operation is large, and the recovery after operation is slow. The simple brachial plexus block cannot effectively meet the operation of shoulder arthroscopy, so nerve block combined with general anesthesia is usually selected for shoulder arthroscopy. According to the analysis of anatomical position I of shoulder arthroscopic surgery, it is concluded that the scope of superior trunk of brachial plexus block (STBPB) combined with superior cervical plexus block (SCPB) is perfect and more suitable for its surgical operation. However, simple brachial plexus superior trunk combined with superficial cervical plexus block cannot completely reduce the pain of patients, and compound general anesthesia is an excellent supplement [21].

Visual anesthesia methods, especially ultrasound imaging, make the operation of nerve block more and more accurate in clinic [22]. The application of ultrasound makes anesthesia develop to visualization. Compared with the positioning of traditional anatomical techniques, nerve block under ultrasound guidance can achieve a perfect effect. Some studies have also shown that compared with the anatomical manual positioning nerve block group, although the operation time of patients in the ultrasound-guided nerve block group is long, the time of pain blocking is shortened and the postoperative analgesia time is prolonged, which improves the satisfaction of patients with the anesthetic effect [23]. Ultrasound-guided nerve block is not only better than anatomical manipulation, but also better than nerve block under the localization of nerve stimulator. Studies have shown that compared with nerve stimulator, ultrasound-guided intermuscular brachial plexus block (ISBPB) can reduce the dosage of local anesthetics and reduce the incidence of intraoperative hypertension. Moreover, ultrasound-guided nerve block can not only reduce the possibility of vascular injury during puncture and improve the safety of anesthesia, but also reduce the use of local anesthetics. Some studies have compared the analgesic effect of ultrasound guidance and nerve stimulator positioning after total knee arthroplasty. The results showed that ultrasound-guided femoral nerve block shortened the operation and onset time, and there were no related complications after nerve block, such as nerve injury and vascular injury. Therefore, ultrasound-guided anesthesia is safer and more effective, not only reducing the incidence of nerve obstruction complications, but also improving patient satisfaction. In arthroscopic shoulder surgery, ultrasound-guided modified upper trunk brachial plexus combined with superficial cervical plexus nerve block has obvious advantages and value [24].

Combining general anesthesia with regional nerve blocks can significantly reduce the incidence of stress and reduce the use of general anesthetic drugs during surgery. Therefore, group A was compared with group C. In shoulder arthroscopy, modified brachial plexus and superficial cervical block combined with ultrasound-guided general anesthesia were used and compared with general anesthesia. There were no significant differences in BMI, operation time, age, or T1 and T2 BIS values between the two groups. Imaging was lower in both groups at 5, 30, and 30 minutes postoperatively due to the use of controlled hypotension. Patients in group C underwent modified brachial plexus superior trunk combined with superficial cervical plexus block, which can effectively block the afferent of noxious stimulation and greatly reduce the dosage of sevoflurane and sufentanil during operation [25].

Ropivacaine is a pure S-type enantiomer with similar chemical structure to bupivacaine. A large number of studies have shown that the anesthetic effect of equal dose ropivacaine is basically the same as that of bupivacaine. Compared with bupivacaine, ropivacaine has the advantages of low toxicity and separation of motor block and sensory block. It is widely used in nerve block anesthesia. Studies have shown that in axillary brachial plexus block, compared with 0.25% and 0.3% ropivacaine, the effect of 0.375% ropivacaine is faster and perfect. Other studies have shown that when performing ultrasound-guided intermuscular sulcus brachial plexus block anesthesia, the application of 30 ml ropivacaine with a concentration of 0.3% ∼ 0.5% can improve the effect of anesthesia block, and the onset speed of anesthesia and the duration of block are positively correlated with the concentration of ropivacaine [26]. Although high concentration of ropivacaine can significantly enhance the blocking effect and prolong the duration of analgesia, when performing intermuscular sulcus brachial plexus block, there is little difference in block time and analgesic duration between 0.375% ropivacaine and 0.5% ropivacaine, and low concentration ropivacaine is helpful in reducing the occurrence of complications such as dizziness, bradycardia, hoarseness, and Horner syndrome. 0.35% ropivacaine was mainly used for nerve block anesthesia [27].

More than 1 million patients worldwide need shoulder arthroscopic surgery every year. Patients undergoing shoulder arthroscopic surgery are often complicated with severe pain, especially within 24 to 48 hours after operation. Severe postoperative pain will limit the patient's activity and is not conducive to the patient's rapid recovery. Long and effective postoperative analgesia can promote the rehabilitation of patients and reduce the length of hospital stay. Therefore, postoperative analgesia is of great significance to patients undergoing shoulder arthroscopy. The traditional method of patient-controlled intravenous analgesia is often used for postoperative analgesia, and opioids are often used. Although the effect of patient-controlled intravenous analgesia is obvious, patients are prone to drug dependence, nausea and vomiting, dizziness, respiratory depression, or skin pruritus and other adverse reactions, causing pain to some patients. Therefore, multiple nerve blocks are performed before shoulder arthroscopic surgery to relieve postoperative pain [28].

Most experts agree that intramuscular tunnel cyanosis is used in combination with general anesthesia for endoscopic shoulder surgery. Compared with patients with general anesthesia, patients with intermuscular bronchial obstruction had more stable intraoperative hemodynamics, less intraoperative anesthesia, and shorter postoperative recovery time. Before the induction of general anesthesia, continuous intermuscular sulcus brachial plexus block guided by ultrasound can not only reduce the intraoperative blood pressure and reduce the dosage of general anesthesia and nitroglycerin, but also help the patients with postoperative analgesia and reduce the incidence of postoperative complications. Compared with the simple intravenous general anesthesia group, MAP and HR in the intermuscular sulcus brachial plexus block combined with intravenous general anesthesia group were significantly reduced, the amount of drugs used during operation was reduced, and the definition of operation field was significantly improved. Compared with traditional patient-controlled intravenous analgesia in shoulder arthroscopic surgery, continuous blockade of the intermuscular tunnel after preoperation provided patients with postoperative analgesia and reduced complications associated with intravenous drugs. Studies have shown that ultrasound-guided intramuscular occlusion combined with general anesthesia can reduce intraoperative systemic blood pressure fluctuations, reduce intraoperative analgesic drug dosage, reduce intraoperative antihypertensive drug use, and relieve postoperative pain, which has been established. Therefore, in the shoulder arthroscopic surgery, the traditional intermuscular sulcus brachial plexus block combined with general anesthesia under the guidance of ultrasound is carried out to explore the advantages and disadvantages from the aspects of intraoperative blood pressure, intraoperative drug dosage, postoperative pain score, postoperative analgesic drug dosage, and postoperative elbow and wrist muscle strength. Compared with patients in group A, patients in group B had better intraoperative blood pressure control, less intraoperative dosage of sufentanil and sevoflurane, lower postoperative pain scores, less postoperative analgesia, and less postoperative nausea and vomiting. However, elbow flexion and wrist muscle strength were significantly reduced after surgery. Patients in group B had complete occlusion of upper limb sensory and motor nerves on the operative side and discomfort and were not suitable for early postoperative shoulder joint rehabilitation training.

Traditional ultrasound blockade of intramuscular cyanosis before general anesthesia can significantly reduce the amount of analgesics during and after shoulder endoscopic surgery and significantly reduce the VAS score after shoulder surgery. It affects the muscle strength of the upper limbs and is usually blocked outside the operation, which cannot achieve the purpose of precise anesthesia and is not conducive to the rapid recovery of patients. To investigate a more accurate method of nerve occlusion, Teha et al. compared shoulder muscle arthroscopy with shoulder arthroscopy and concluded that cranial tubercle occlusion can achieve the same results as anesthesia. The better the motor block, the lower the incidence of Horner syndrome; however, when the supraclavicular bronchial obstruction was performed, local anesthetic penetrated the upper, middle, and lower trunks of the intervertebral disc, and there was no significant difference in muscle strength.

Shalini et al. found that patients with suprascapular and axillary nerve block combined with general anesthesia had lower 24-hour postoperative pain scores than the intramuscular brachial plexus block combined with general anesthesia group; therefore, capillary and axillary nerve occlusion during shoulder endoscopic surgery combined with general anesthesia may help relieve long-term postoperative pain. In addition, suprascapular joint axillary nerve blocks are used for postoperative pain relief with slightly different pain levels. Patients undergoing shoulder arthroscopy were more likely to receive a suprascapular axillary nerve block for postoperative pain relief. Arthroscopic suprascapular joint nerve occlusion surgery usually requires the surgical insertion of more than two needles, which increases the patient's psychological burden and tension and has no obvious advantages compared with intermuscular tunnel obstruction. Shen et al. argued that, compared with the brachial plexus block in the myenteric groove, the C5 nerve root block not only has the same anesthetic effect, but also greatly reduces the incidence of nerve block complications and unnecessary regional blocks. Shoulder arthroscopic surgery was randomly divided into two groups: selective cervical nerve root block (C5, C6 nerve root implantation under 5 ml local anesthetic) and intermuscular block (10ml of local anesthetic was injected with peribrachial plexus). The study showed that the onset time of anesthesia in the cervical nerve root selective block group was shorter than that of the intermuscular inhibition group, and the VAS score at 12 hours after surgery and tramadol dose at 24 hours after surgery were significantly reduced. At 4 hours postoperatively, the radial artery motor score increased significantly.

Although selective nerve root block has little effect on muscle strength, the scope of block is not perfect. According to the anatomical position of shoulder arthroscopy, the nerves to be blocked are supraclavicular nerve, axillary nerve, subscapular nerve, suprascapular nerve, and musculocutaneous nerve. The supraclavicular nerve is the branch of the nerve originating from the superficial cervical junction, and the remaining four nerves are the main branches of the upper breast; therefore, shoulder arthroscopy will examine the cervical tubercle and superficial cervical occlusions relative to traditional trunk and superficial cervical occlusions, where the intercostal space has been modified to take advantage of general anesthesia. When the modified upper trunk of brachial plexus and superficial cervical plexus nerve blocks are performed under the guidance of ultrasound, one-needle operation is often used, that is, one needle is inserted and gradually blocked, which relives the psychological burden and tension of patients during nerve operation. Compared with group C, group B showed that PACU, elbow, and wrist flexion increased significantly at 6 h after operation, and the amount of sevoflurane during operation was significantly reduced. Compared with traditional interstitial cyanosis and cervical tubercle occlusion changes, it has less effect on elbow muscle strength, less impact on wrist muscle strength, low intraoperative anesthesia, and low postoperative incidence. The incidence of postoperative nausea and vomiting nerve block related complications was low; the advantages of small influence on muscle strength are conducive to reducing postoperative discomfort of patients, contributing to early functional exercise of patients, so that patients get early recovery. Moreover, the reduction of intraoperative sevoflurane dosage can shorten patient resuscitation time, making the hemodynamics more stable during surgery.

## 5. Conclusion

Ultrasound has been shown to improve the depth of anesthesia during surgery compared to conventional intramuscular block combined with general anesthesia in shoulder surgery. Furthermore, it reduces the doses of controlled hypotension, postoperative anesthetics, and postoperative analgesics; reduces postoperative pain; and reduces the incidence of postoperative side effects. In addition, it has little effect on the strength of the elbow and wrist flexors, which is more conducive to the early recovery of patients. This suggests that the use of ultrasound to block the upper part of the breast during shoulder surgery can effectively resolve postoperative pain, compensate for unbearable pain after surgery, and improve the patient's ability to recover.

## Figures and Tables

**Figure 1:** Shoulder joint diagram.

**Figure 2:** MAP changes of patients in each group.

**Figure 3:** HR changes of patients in each group.

**Table 1:** Comparison of general information and BIS value of patients in each group.

Group	Quantity	Age	BMI	Operation time (min)	BIS value of T1	BIS value of T2
A	30	59.90 ± 5.84	23.44 ± 2.47	59.07 ± 12.77	51.40 ± 4.32	51.00 ± 4.38
B	30	58.63 ± 6.70	24.17 ± 3.13	59.90 ± 11.21	50.53 ± 3.78	51.70 ± 2.59
C	30	60.10 ± 6.78	22.99 ± 2.21	55.33 ± 14.11	52.17 ± 4.42	52.37 ± 2.19

**Table 2:** MAP changes of patients in each group.

Group	T0	T1	T2	T3
A	97.00 ± 7.10	86.87 ± 4.49	76.97 ± 8.14	104.60 ± 7.11
B	95.93 ± 7.22	67.90 ± 6.23	67.80 ± 6.19	94.73 ± 8.46
C	97.77 ± 6.40	66.90 ± 4.81	66.63 ± 4.81	92.43 ± 7.32

**Table 3:** HR changes of patients in each group.

Group	T0	T1	T2	T3
A	72.70 ± 5.13	62.70 ± 8.91	63.73 ± 8.71	75.00 ± 9.45
B	71.01 ± 8.64	54.80 ± 4.43	54.30 ± 4.44	64.63 ± 8.47
C	70.83 ± 7.71	55.60 ± 5.91	55.67 ± 5.49	68.47 ± 8.98

## Data Availability

The data used to support the findings of this study are available from the corresponding author upon request.

## References

[1] Druzhinin V. N., Suvorov V. G., Shelekhova A. E. (2020). Optical density of bone tissue in the dynamics of therapy of professionally caused osteopathies of the shoulder joint. *Russian Journal of Occupational Health and Industrial Ecology*.

[2] Strafun S. S., Serhienko R. A., Nehria N. M. (2020). The role of the biceps tendon instability in the development of rotator cuff arthropathy of the shoulder joint. *Trauma*.

[3] K C. K., L R. A., V G. T., M P. S. (2020). Intrarater and interrater reliability of timed functional arm and shoulder test in patients with shoulder joint pathology-a cross-sectional study. *International Journal of Scientific and Research Publications (IJSRP)*.

[4] Tregubova E. S., Kozlova N. S. (2020). Pathogenesis of post-stroke periarthropathy of the shoulder joint from the perspective of somatic dysfunctions. *Russian Osteopathic Journal*.

[5] Sahara R., Hamada J., Yoshizaki K., Endo K., Segawa D., Yamaguchi M. (2020). Kinematic differences between two types of forward elevations of the shoulder joint: flexion and reaching elevation. *The Open Orthopaedics Journal*.

[6] Chen G., Cui L., Chen P., Li W., Liu G. (2020). Experimental study on reconstruction of anterior labrum of shoulder joint by chemical extraction of allogeneic tendon and allogeneic chondrocytes. *Zhongguo xiu fu chong jian wai ke za zhi = Zhongguo xiufu chongjian waike zazhi = Chinese journal of reparative and reconstructive surgery*.

[7] Yakovenko S., Kotulskiy I., Petrova I. (2020). Ultrasonographic features in pathological changes of shoulder joint’s periarticular tissues in patients with different manifestations of pain syndrome. *Orthopaedics, Traumatology and Prosthetics*.

[8] Qiang L., Xi X.-K., Xiao T., Hou J.-P., Qi W.-W., Wang K.-N. (2022). Design and research of an electric shoulder joint harmonic reducer for a moving and lifting exoskeleton robot. *Journal of King Saud University - Engineering Sciences*.

[9] Lee K. (2021). An abrupt-onset shoulder joint subluxation and pseudoparalysis caused by intraarticular pigmented villonodular synovitis: a case report. *Joint Diseases and Related Surgery*.

[10] Meder A., Stefanescu M. C., Ateschrang A. (2021). Evidence-based examination techniques for the shoulder joint. *Zeitschrift fur Orthopadie und Unfallchirurgie*.

[11] Nikolaev N. S., Alekseeva A. V., Yakovlev V. N., Lushin A. V. (2021). The effectiveness of current methods of surgical treatment of anterior recurrent instability of the shoulder joint, depending on anatomical and functional changes. *Genij Ortopedii*.

[12] Chen S., Yan Y., Xu G., Gao X., Tai C. (2021). Mirror-type rehabilitation training with dynamic adjustment and assistance for shoulder joint. *Sheng wu yi xue gong cheng xue za zhi = Journal of biomedical engineering = Shengwu yixue gongchengxue zazhi*.

[13] Chen S., Shi Y., Xue P., Chen X. (2021). Application value of magnetic resonance arthrography of the shoulder in nursing and diagnosis of patients with shoulder joint injury. *Journal of Healthcare Engineering*.

[14] Summers T. K., Sookhoo B. D., Stumpo L., Parada S. A. (2020). Suprascapular artery aneurysm secondary to severe shoulder joint osteoarthritis. *Case Reports in Orthopedic Research*.

[15] Varghese R. J., Lo B., Yang G. Z. (2020). Design and prototyping of a bio-inspired kinematic sensing suit for the shoulder joint: precursor to a multi-dof shoulder exosuit. *IEEE Robotics and Automation Letters*.

[16] Galluccio F., Fajardo Perez M., Yamak Altinpulluk E., Hou J.-D., Lin J.-A. (2021). Evaluation of interfascial plane and pericapsular nerve blocks to the shoulder joint: a preliminary analysis of shoulder anterior capsular block. *Pain and Therapy*.

[17] Engelkes K., Panpeng S., Haas A. (2021). Ontogenetic development of the shoulder joint muscles in frogs (amphibia: anura) assessed by digital dissection with implications for interspecific muscle homologies and nomenclature. *Zoomorphology*.

[18] Ru O. A., Xl B., Rui W. B., Qz A., Ys B., El A. (2020). Effect of ultrasound-guided right stellate ganglion block on perioperative atrial fibrillation in patients undergoing lung lobectomy: a randomized controlled trial - sciencedirect. *Brazilian Journal of Anesthesiology (English Edition)*.

[19] Sundaram S., Dhakshinamoorthy M., Swaminathan G. A. (2020). Observational study on the accuracy and speed of ultrasound guided transversus abdominis plane block with two different monitor positions. *Indian Journal of Clinical Anaesthesia*.

[20] Wang J., Lu Y. (2020). Application of ultrasound-guided bilateral erector spinae plane block in lumbar spinal surgery. *Annals of Palliative Medicine*.

[21] Gelber J., Luftig J., Mantuani D. (2021). Ultrasound-guided retroclavicular approach to the infraclavicular region (RAPTIR) anesthesia for challenging upper extremity reductions. *Journal of Emergency Medicine*.

[22] Fan M., Sharma A. (2021). Design and implementation of construction cost prediction model based on svm and lssvm in industries 4.0. *International Journal of Intelligent Computing and Cybernetics*.

[23] Liu X., Liu J., Chen J., Zhong F., Ma C. (2021). Study on treatment of printing and dyeing waste gas in the atmosphere with Ce-Mn/GF catalyst. *Arabian Journal of sciences*.

[24] Yuvaraj N., Srihari K., Dhiman G. (2021). Nature-inspired-based approach for automated cyberbullying classification on multimedia social networking. *Mathematical Problems in Engineering*.

[25] Shriram S., Jaya J., Shankar S., Ajay P. (2021). Deep learning-based real-time AI virtual mouse system using computer vision to avoid COVID-19 spread. *Journal of Healthcare Engineering*.

[26] Nsm A., Nra B., Dp C., Bo A., Cf A., Acc A. (2020). Efficacy of ultrasound guided suprascapular block in patients with chronic shoulder pain: observational, retrospective study - sciencedirect. *Brazilian Journal of Anesthesiology (English Edition)*.

[27] Huang R., Zhang S., Zhang W., Yang X. (2021). Progress of zinc oxide‐based nanocomposites in the textile industry. *IET Collaborative Intelligent Manufacturing*.

[28] Merella F., Mossetti V. (2020). Ultrasound-guided upper and lower extremity nerve blocks in children. *BJA Education*.

